This article has been retracted.

# Network Management System for IoT Based on Dynamic Systems

**DOI:** 10.1155/2021/9102095

**Published:** 2021-12-13

**Authors:** Mohammad Alsaffar, Abdulsattar Abdullah Hamad, Abdullah Alshammari, Gharbi Alshammari, Tariq S. Almurayziq, Mohammed Shareef Mohammed, Wegayehu Enbeyle

**Affiliations:** ^1^College of Computer Science and Engineering, Department of Computer Science and Information, University of Ha'il, Saudi Arabia; ^2^College of Sciences, Department of Mathematics and Computer Sciences, Tikrit University, Iraq; ^3^Ministry of Education, Iraq; ^4^Department of Statistics, Mizan-Tepi University, Ethiopia

## Abstract

The Internet of Things (IoT) has the potential to transform the public sector by combining the leading technical and business trends of mobility, automation, and data analysis to dramatically alter the way public bodies collect data and information. Embedded sensors, actuators, and other devices that capture and transmit information about network activity in real-time are used in the Internet of Things to connect networks of physical objects. The design of a network management system for an IoT network is presented in this paper, which uses the edge computing model. This design is based on the Internet management model, which uses the SNMP protocol to communicate between managed devices, and a gateway, which uses the SOAP protocol to communicate with a management application. This work allowed for the identification and analysis of the primary network management system initiatives for IoT networks, in which there are four fundamental device management requirements for any deployment of IoT devices: provisioning and authentication, configuration and control, monitoring and diagnostics, and software updates and maintenance.

## 1. Introduction

A wide variety of devices make up computer networks. They want to facilitate communication and resource sharing. The efficiency of the services provided is linked to the network's systems' performance to a large extent. The management of computer networks arose due to the rapid evolution of network technologies, which was accompanied by a significant decrease in the cost of computing resources [1]. We have now arrived at the Internet of Things (IoT) from simple resource sharing to much more complex applications such as email, file transfer, and multimedia applications, and we have now arrived at the Internet of Things (IoT). [2] look at two key aspects of the Internet of Things: technological advancements in remote connectivity and the potential commercial implications of product digitization. They conclude that the Internet of Things is not a single concept or paradigm but rather a collection of options from which each actor can choose the best approach for its strategic goals and commercial needs.

Specific areas of the industry, such as health, home, and transportation, have developed IoT advancements, resulting in the creation of various architectures and management mechanisms, which are made up of technologies, protocols, and different standards. It is important to remember that traditional network management models (OSI, ITU, and Internet) were created assuming that the devices being managed have adequate processing and communication capabilities. This is not the case in the IoT world, as many devices have limited processing, storage, and connectivity capabilities, necessitating proper configuration and updating of the applications running on them in order for them to function properly. Various studies for the implementation of IoT management have been developed based on the preceding. According to Prince et al. [3], four trends in IoT management implementation are classified based on the management mechanism or standard used: SNMP, TMN, WBEM, and PBM. Because of the widespread adoption of SNMP among manufacturers, it is the most appealing standard for IoT management implementation. Several studies have been conducted in recent years with the goal of adapting this protocol to an IoT network. Jungyoung et al. [4] describe an SNMP-based IoT management method and the configuration of the MIB, agent, and management application. The agent saves all of its information in a tree of MIBs, containing variables containing the values representing the sensor data. To know the information of the sensor, the management application can send a message to the agent of the managed IoT devices with sensors and obtain the value of the variables stored in MIB.

On the other hand, management based on PBM entails employing autonomous management, which is achieved through the fulfillment of four functionalities: self-configuration, self-repair, self-optimization, and self-protection. As a result, this type of management stands out for altering the role of the operator, who now performs functions associated with policy definition rather than directly controlling the system. Finally, it is worth mentioning that cloud service platforms have their management models. This is the case with Azure IoT Hub [5], a cloud-based managed service that serves as a message center for two-way communications between IoT applications and the devices they manage. It has features and an extensibility model that allow device and back-end developers to create robust device management solutions [6]. Device management patterns such as reboot, factory reset, configuration, firmware update, and status and progress reports are available through Azure IoT Hub [7–12]. IoT has yet to see the development of a standardized autonomous management system [13–15]. Only a few software proposals in specific areas of the autonomous management system are highlighted. In light of the foregoing, this document presents a network management system design for an IoT network based on the edge computing model, which allows for efficient monitoring and configuration.

## 2. Specification and Design of the Network Management System Architecture

This research aims to design, using the edge computing model, a network management system for an IoT network that allows monitoring and configuration, as well as to implement a prototype that allows validating the design. Based on the above, the conditions for the architecture design and management functions are presented below.

### 2.1. Architecture Design and Management Functions

The network management system is designed with the three components of the computing model at the edge in mind, namely, the IoT devices, [4, 16–20] the IoT Gateway, and the cloud Figure 1, and development of the network management system implies the definition of aspects related to the information of the IoT devices to be managed, precisely the attributes.

Given that a standard network management architecture had to be chosen, the following three options were considered:

- OSI management model
- ITU management model
- Model for internet management. It is important to note that the communication protocol used in the OSI and ITU models is CMIP, whereas the one used in the Internet model is SNMP. As a result, the selection was primarily based on the communication protocol and the information structure associated with each one

The selection of the Internet management model to implement the IoT network management system was based on the simplicity and low memory and resource use of the SNMP protocol, which is one of the main characteristics of IoT devices, as compared to the CMIP protocol used in the OSI and ITU management models. Similarly, even though SNMP does not natively support task execution, some implementations do, based on the definition of information objects developed for this purpose (Table 1).

In contrast, version 2c was chosen for the SNMP version because it is the most widely used and because its functionalities enable the implementation of an IoT network management system. However, version 3, which provides improved security options for the SNMP protocol, may be considered in future versions. The Internet management model specifies an information structure in which OID, and information bases are used management MIB, of which some are standard types. However, given the characteristics of IoT devices and the applications they support, which are primarily based on sensors, a private MIB with specific information on said devices was designed, which is not included in standard type MIBs. This MIB's function is to deliver information about the status of various sensors on the IoT device. Based on the preceding, the structure of the private MIB for IoT is depicted in Figure 2.

Table 2 describes the objects of the IoT sensor subtree, which is based on the MIB-II interface group.

Likewise, Tables 2 and 3 show the description of the objects of the IoT software subtree, used for updating the IoT devices, and which is based on the Cisco OLD-CISCO-FLASH-MIB MIB.

Additionally, other information objects are included, related to other functions, or observed in Table 3. Finally, for the management of failures in IoT devices, the counter traps are included in Table 4.

Communication between the IoT Gateway and the management application must allow data exchange between the two nodes and file exchange to send software updates to the devices via this medium. IoT.

In the context of IoT, numerous protocols allow data to be exchanged between devices and the cloud.  Table 5 compares the options considered, with SOAP being chosen primarily for the security features it provides.

### 2.2. Design of the IoT Device Agent

Taking into account the management functions in the IoT device, the design developed for the agent is made up of 4 modules, as can be seen in Figure 3.

The Internet of Things (IoT) has the potential to transform the public sector by combining the main technical and business trends of mobility, automation, and data analysis to alter the way public bodies collect data and information dramatically. Embedded sensors, actuators, and other devices that capture and transmit information about network activity in real time are used in the Internet of Things to connect networks of physical objects. The design of a network management system for an IoT network is presented in this paper, which uses the edge computing model. This design is based on the Internet management model, which uses the SNMP protocol to communicate between managed devices and a gateway, which uses the SOAP protocol to communicate with a management application. This work allowed for the identification and analysis of the main network management system initiatives for IoT networks, in which there are four fundamental device management requirements for any deployment of IoT devices: provisioning and authentication, configuration and control, monitoring and diagnostics, and software updates and maintenance.

### 2.3. Design of the IoT Gateway Manager

Considering the management functions in the IoT Gateway, the manager is made up of 5 modules, as shown in Figure 4.

The “SNMP manager” module implements the functionalities of the SNMP protocol, from the manager's point of view, which, as previously indicated, corresponds to version 2c, taking into account that version 3 can later be implemented.

The “IoT device monitoring” module is in charge of monitoring the status of IoT devices, that is, whether they are available or not. The “SOAP agent” module is responsible for communicating between the IoT gateway and the management application through the SOAP protocol. The “software distribution” module is responsible for distributing the update software to IoT devices.

Finally, the “administration” module allows remote configuration of the IoT gateway, by accessing and modifying the configuration database.

### 2.4. Design of the Cloud Computing Platform Management Application

Taking into account the management functions in the management application, it is made up of 4 modules, as can be seen in Figure 5.

The “SOAP agent” module uses the SOAP protocol to communicate between the management application and the IoT gateway. The “Gateway IoT monitoring” module is responsible for keeping track of the status of IoT gateways. The “software distribution” module is in charge of sending update software to IoT devices. It interacts with the “SOAP Agent” module to send the update software to the IoT gateway for the purposes stated above. Finally, the “administration” module allows for remote configuration of the cloud management application's parameters, which are saved in a database. Similarly, information on IoT devices sent by IoT gateways is displayed and modified via a web interface through this module.

## 3. Conclusions

The network management system's architecture design enables the devices deployed in an IoT network to be managed simply. The information object model's structure enables the management of data from IoT device sensors straightforwardly.

On the other hand, the specification and design of the architecture of an IoT networks network management system under the edge computing model, including its elements: IoT device, IoT gateway, and cloud, were completed. This design enables simple management of devices deployed in an IoT network. The information object model's structure enables the management of data from IoT device sensors straightforwardly.

It is important to remember that in scenarios with thousands of IoT devices, transfer rates can be hampered if their monitoring timers are not properly configured, that is, if they are set to very low values, even though these devices send heartbeat messages to the IoT gateway regularly. Similarly, IoT devices can be continuously detected as unavailable by the IoT gateway in unstable local networks, affecting the transfer rates between this element and the management application because SOAP messages informing about these state changes would be sent constantly.

Despite the fact that the developed design only took into account sensor characteristics associated with their states (administrative and operational), the proposed structure of information objects allows for future addition of additional sensor or IoT device characteristics, such as those related to energy consumption.

On the other hand, the heterogeneity of the characteristics of the devices and sensors on the market can be homogenized through a well-designed network management system, such as standardizing the way of querying the status (administrative and operational) of the sensors to make their management tasks easier. However, this necessitates the creation of a unique driver for each sensor.

The IoT gateway is a critical component of the edge computing model. This element is given special attention in the developed design because it is the one that performs continuous monitoring of IoT devices, increasing the management system's reliability by removing the reliance on cloud connections.

Incorporating protocols such as SNMP and SOAP into the design makes it possible to support the standardization process, as these are currently widely used in the industry.

In terms of the implemented prototype, it allowed for the validation of the operation of the designed characteristics using a test protocol created specifically for this purpose. Given that the implementation was mostly done in Java, it could be evaluated in the future using C, specifically for the IoT device and the IoT gateway.

Companies that have implemented a network of IoT devices and require a tool to manage them are potential users of the implemented prototype.

Finally, the implementation of SNMP v3 at the communication level between the IoT device and the IoT gateway may be related to future developments in the designed network management system. Similarly, even though SOAP was chosen as the communication protocol between the IoT gateway and the management application, additional protocols such as REST could be implemented, allowing the user to choose based on the performance characteristics they require in a specific way.

## Figures and Tables

**Figure 1:** Components of the IoT device management system.

**Figure 2:** Structure of the management system.

**Figure 3:** Components of the IoT.

**Figure 4:** Components of the IoT manager.

**Figure 5:** Components of the cloud management application.

**Table 1:** Attribute comparison between SNMP and CMIP.

Attribute	SNMP	CMIP
Deployment simplicity	Yes (+)	Not natively (+)
Resource consumption	No (-)	Not natively (-)
Performing tasks	Not natively (+)	Yes (+)
File transfer	Not natively (+)	Yes (+)

**Table 2:** Sensor subtree objects.

Object	Description	Syntax	Permission
sNumber	Number of sensors in the IoT device	Integer	Read only
sTable	List of sensors present in the device	Sequence of sEntry	Not accessible
sEntry	Input containing information from a sensor	sEntry	Not accessible
sIndex	Contains sensor information/sensor type	Integer	Read only
sDescr	Sensor operation configured status	DisplayString	Read only

sType	Sensor type	Integer {	Read only
		List of sensor types}	

sStatusAdmin	Sensor operation configured status	IInteger {	Read and write
		Up (1)	
		Down (2)}	

sOperator status	Current status of sensor operation	Integer {	Read only
		Up (1)	
		Down (2)}	

**Table 3:** IOT software subtree objects and información objetos.

Object	Description	Syntax	Permission
swVersion	Current version of IoT device software	DisplayString	Read only
swTo update	Name of the software version to download from the file server	DisplayString	Write only
swUpdate status	Status of the current or last update	Integer {in progress (1), success (2), fail (3), and noAfterPowerOn (4)}	Read only
swUpdate date	Date of last update	DisplayString	Read only

Designed traps			
Heartbeat	Other information objects		
	The IoT device sends a heartbeat to the IoT gateway	Integer	Read only

**Table 4:** Designed traps.

Object	Description	Syntax
Heartbeat	Indicates that the agent is available. The sending time of this trap is configured in the OID heartbeat (1.3.6.1.4.1.50000.3.1)	1.3.6.1.6.3.1.1.5.50000.1
sensorDown admin	Indicates that the agent has detected that the sensor has changed its administrative state to OFF. The value of this trap indicates the affected sensor.	1.3.6.1.6.3.1.1.5.50000.2
sensorUp admin	Indicates that the agent has detected that the sensor has changed its administrative state to ON. The value of this trap indicates the affected sensor.	1.3.6.1.6.3.1.1.5.50000.3
sensorDown operator	This indicates that the agent has detected that the sensor has changed its operational state to OFF. The value of this trap indicates the affected sensor.	1.3.6.1.6.3.1.1.5.50000.4
sensorUp operator	Indicates that the agent has detected that the sensor has changed its operational state to ON. The value of this trap indicates the affected sensor.	1.3.6.1.6.3.1.1.5.50000.5
Upgrade	Indicates that the IoT device has finished updating the software. The value of this trap indicates the result of this process, in accordance with those indicated in the OID sw update status (1.3.6.1.4.1.50000.2.3), which can be successful (2) or failure (3). The result can also be consulted through the mentioned OID.	1.3.6.1.6.3.1.1.5.50000.6

**Table 5:** Comparison of communication options between IoT and the management app.

Attribute	MQTT	SOAP	REST
Allows data exchange	Yes	Yes	Yes
Allows file sharing	No	Yes	Yes
Resource consumption	Low	High	Half
Security measures	Medium (SSL/TLS)	High (WS-security and SSL/TLS)	Medium (SSL/TLS)

## Data Availability

The data underlying the results presented in the study are available within the manuscript.
